RETRACTED

# Multimodal MRI-Based Radiomic Nomogram for the Early Differentiation of Recurrence and Pseudoprogression of High-Grade Glioma

**DOI:** 10.1155/2022/4667117

**Published:** 2022-09-30

**Authors:** Hui Jing, Fan Yang, Kun Peng, Danlei Qin, Yexin He, Guoqiang Yang, Hui Zhang

**Affiliations:** ^1^College of Medical Imaging, Shanxi Medical University, Taiyuan, Shanxi Province, China; ^2^Department of Radiology, The Sixth Hospital, Shanxi Medical University, Taiyuan, Shanxi Province, China; ^3^Department of Radiology, Shanxi Provincial People's Hospital, Affiliated People's Hospital of Shanxi Medical University, Taiyuan, China; ^4^Department of Radiology, First Clinical Medical College, Shanxi Medical University, Taiyuan, Shanxi Province, China; ^5^Shanxi Key Laboratory of Intelligent Imaging and Nanomedicine, Shanxi Medical University, Taiyuan, Shanxi Province, China

## Abstract

**Objective:**

To evaluate the diagnostic value of multimodal MRI radiomics based on T2-weighted fluid attenuated inversion recovery imaging (T2WI-FLAIR) combined with T1-weighted contrast enhanced imaging (T1WI-CE) in the early differentiation of high-grade glioma recurrence from pseudoprogression.

**Methods:**

A total of one hundred eighteen patients with brain gliomas who were diagnosed from March 2014 to April 2020 were retrospectively analyzed. According to the clinical characteristics, the patients were randomly split into a training group (*n* = 83) and a test group (*n* = 35) at a 7 : 3 ratio. The region of interest (ROI) was delineated, and 2632 radiomic features were extracted. We used multiple logistic regression to establish a classification model, including the *T*1 model, *T*2 model, and *T*1 + *T*2 model, to differentiate recurrence from pseudoprogression. The diagnostic efficiency of the model was evaluated by calculating the area under the receiver operating characteristic curve (AUC) and accuracy (ACC) and by analyzing the calibration curve of the nomogram and decision curve.

**Results:**

There were 75 cases of recurrence and 43 cases of pseudoprogression. The diagnostic efficacies of the multimodal MRI-based radiomic model were relatively high. The AUC values and ACC of the training group were 0.831 and 77.11%, respectively, and the AUC values and ACC of the test group were 0.829 and 88.57%, respectively. The calibration curve of the nomogram showed that the discrimination probability was consistent with the actual occurrence in the training group, and the discrimination probability was roughly the same as the actual occurrence in the test group. In the decision curve analysis, the *T*1 + *T*2 model showed greater overall net efficiency.

**Conclusion:**

The multimodal MRI radiomic model has relatively high efficiency in the early differentiation of recurrence from pseudoprogression, and it could be helpful for clinicians in devising correct treatment plans so that patients can be treated in a timely and accurate manner.

RETRACTED

## 1. Introduction

Glioma is the most common primary malignant tumor of the central nervous system, accounting for approximately 50% of all primary malignant tumors, and it has high disability and mortality rates [1, 2]. It has been reported that the median survival time of glioblastoma patients is only 15 months, and the two-year survival rate is less than 30% [3]. Second, because of its strong invasive growth characteristics, the tumor tissue cannot be completely removed by surgery, and maximum surgical resection and postoperative adjuvant radiotherapy and chemotherapy are needed to delay the time until recurrence. Surgical resection plus postoperative radiotherapy or combined radiotherapy and chemotherapy has become the most important methods for the treatment of gliomas [4]. However, new enhanced lesions sometimes appear in the treatment area on MRI images after treatment with radiotherapy or after treatment that combines radiotherapy and chemotherapy, and these new lesions can be due to recurrence or pseudoprogression of the tumor [5]. Recurrence is due to the continuous proliferation of the tumor blood vessels, a large increase in the number of tumor cells, and continuous infiltration of the surrounding normal brain parenchyma, eventually leading to the destruction of the blood-brain barrier. Pseudoprogression is defined as local inflammation, edema, a transient increase in blood-brain barrier permeability and injury of oligodendrocytes caused by radiotherapy and chemotherapy, and pseudoprogression mostly occurs 3-6 months after surgery [6]. Clinically, the treatment schemes of these two phenomena are completely different. There can be a good prognosis in pseudoprogression even without invasive treatment interventions, while patients with recurrence must be treated in time to delay further development of the disease. Therefore, the accurate differentiation of these two phenomena is very important for patients with intracranial gliomas.

According to the response assessment in neuro-oncology (RANO), the commonly used methods that distinguish the two are secondary postoperative pathology or a long-term follow-up of more than 6 months [7]. Histopathology is currently recognized as the gold standard, but it is an invasive examination with many limitations, while long-term follow-up of more than 6 months is relatively long, which can lead to a delay in treatment. Therefore, it is crucial to seek a simple, effective, and early method to distinguish recurrence from pseudoprogression of a glioma.

RETRACTED

As a new method of data processing and image analysis, radiomics can obtain image features that cannot be directly recognized only by direct human vision on medical images and can mine information about the tumor grade, genetics, curative effect, and prognosis that are contained in the imaging data. Radiomics can express the characteristics of postoperative changes in gliomas at multiple levels, comprehensively guide early diagnosis and middle-term treatment, and evaluate the prognosis of glioma [8–10]. Jang et al. [11] proposed machine learning methods based on MRI imaging to identify pseudoprogression and recurrence of glioblastomas. Kocher et al. [12] proposed radiomic and machine learning methods based on MRI and PET to distinguish the recurrence and pseudoprogression of malignant brain tumors. Currently, most hospitals conduct plain and enhanced MRI scans for the diagnosis or reexamination of gliomas. Therefore, this study explored the value of multimodal MRI radiomics based on T2WI-FLAIR combined with T1WI-CE images for the early differential diagnosis of recurrence versus pseudoprogression. This study provides a basis for obtaining early, accurate diagnosis and treatment and has important clinical application value.

## 2. Materials and Methods

The experiment used a retrospective design and was approved by the Shanxi Medical University ethics committee (2019LL101), and the informed consent requirement was waived due to the retrospective study design.

### 2.1. Patients

A total of one hundred eighteen patients with brain gliomas that were confirmed in two centers from March 2014 to April 2020 were analyzed retrospectively. All patients had new enhanced lesions or enlarged enhancement areas on their second MRI reexamination, which was performed within 1-3 months. Among all of the patients, there were 72 men and 46 women, and they were aged from 12 to 82 years old, with an average age of 50.24 ± 14.27 years old. The inclusion criteria were (1) high-grade gliomas were confirmed by neurosurgery and pathology (grades III and IV according to the WHO CNS 2007 standards for classification); (2) the patient had postoperative adjuvant radiotherapy and chemotherapy; (3) the plain and enhanced MRI scans performed within 2 days after surgery were the baseline images; (4) a second MRI reexamination at 1-3 months found new enhanced lesions or an enlarged enhancement range; (5) the patient's Karnofsky score (Karnofsky Performance Status, KPS) was 70-90, and the patient's median KPS score was 80; and (6) the patients with pseudoprogression or recurrence were confirmed by a second operation and via pathology or via a follow-up of more than 6 months. The exclusion criteria were (1) the low-grade gliomas were confirmed by neurosurgery and pathology (grades I and II according to the WHO CNS 2007 standard for classification); (2) the patients did not receive postoperative adjuvant radiotherapy and chemotherapy; (3) the patients' images were not clear; and (4) there were no significant changes in the intracranial lesions during the 1-3 months of follow-up. There were 17 cases of recurrence and 8 cases of pseudoprogression, as confirmed by secondary surgical pathology. 58 cases of recurrence and 35 cases of pseudoprogression were confirmed by long-term follow-up. According to the clinical characteristics, 118 patients were randomly divided into a training group (*n* = 83) and a test group (*n* = 35) at a 7 : 3 ratio and then checked to determine whether there was a significant difference in clinical characteristics between the training group and test group. If there was a significant difference, then, the data were split again until there was no difference in any clinical characteristics between the training group and test group.

RETRACTED

### 2.2. Imaging Sequences, Parameters, and Image Preprocessing

In this study, all patients were examined on a Siemens Avanto 1.5-T and GE HDxt 3.0-T superconductive MRI scanner using a phased array head coil. All images were calibrated, and the scanning parameters were consistent. The scanning parameters of all sequences were as follows: (1) axial T1WI: TE 15 ms, TR 300 ms, FOV 24 cm × 24 cm, matrix size 256 × 256, layer thickness 5 mm, layer spacing 2.5 mm, and NEX 3; (2) axial T2WI: TE 150 ms, TR 3500 ms, FOV 24 cm × 24 cm, matrix size 390 × 390, layer thickness 5 mm, layer spacing 2.5 mm, and NEX 3; (3) axial T2WI-FLAIR: TE 200 ms, TR 5500 ms FOV 24 cm × 24 cm, matrix size 512 × 512, layer thickness 5 mm, layer spacing 2.5 mm, and NEX 3; (4) sagittal T1WI: TE 30 ms, TR 250 ms, FOV 26 cm × 26 cm, matrix size 512 × 512, layer thickness 5 mm, layer spacing 2 mm, and NEX 3; and (5) gadolinium diamine or gadolinium meglumine (Gd-DTPA-BMA or Gd-DTPA) was injected into the anterior elbow vein through an intravenous indwelling needle at a dose of 0.2 ml/kg and at a flow rate of 2 ml/s, and axial TIWI contrast enhanced (T1WI-CE) images were obtained (the scanning parameters were the same as the axial T1WI plain scanning).

The image preprocessing steps were (1) noise reduction, which was achieved by image filtering and the image enhancement technology of the in-house MATLAB software; and (2) registration, in which the T1WI-CE sequence was registered with the T2WI-FLAIR sequence using the General Registration BRAINS function of 3D-Slicer.

RETRACTED

### 2.3. Image Diagnosis and Region of Interest Segmentation

The MRI plain scans and enhanced scans were performed within 48 h after surgery as the baseline images. The second MRI reexaminations at 1-3 months showed whether there were new enhancement lesions or enlargements of the enhancement ranges on the T1WI-CE images. After the secondary postoperative pathology results were obtained or after a long-term follow-up of more than 6 months, the follow-up images were independently diagnosed by two radiologists with intermediate certificates (with 6 years and 8 years of working experience, respectively). The final result was the consensus of the two radiologists' interpretations. When there was a different opinion between the two, the diagnosis was made by a third radiologist with a senior professional title (with 15 years of working experience), and the result was the final diagnosis. A flowchart of the radiomics process for the prediction of recurrence and pseudoprogression of gliomas is shown in Figure 1.

For ROI segmentation, ITK-SNAP software (http://www.itksnap.org) was used to outline the enhanced part of the T1WI-CE images, and the lesions on the T2WI-FLAIR images were outlined based on the T1WI-CE enhanced sequence, which was the region of interest. This ROI was sketched manually by a qualified radiologist and was then checked layer by layer by a senior physician. To maintain the accuracy and consistency of the data, all delineated areas avoided any lesions or artifacts, such as cystic degeneration, necrosis, and blood vessel calcification. The preoperative examination, postoperative follow-up, ROI segmentation, and secondary postoperative pathological images of any recurrence and pseudoprogression of the gliomas are presented in Figures 2–5.

### 2.4. Feature Extraction and Selection

After the images were standardized, the radiomic features were extracted by FAE analysis software (FeAture Explorer, Shanghai Key Laboratory of Magnetic Resonance, East China Normal University), including the first-order intensity features, shape features, texture features, and wavelet features. The synthetic minority oversampling technique (SMOTE) [13, 14] and upsampling algorithms were used to balance the positive and negative sample data in the dataset. SMOTE could not directly resample a small number of classes but designed an algorithm to artificially synthesize some new minority samples. Upsampling increased the number of samples by repeating the evaluation in random cases to achieve a balance between positive and negative samples. The SMOTE and upsampling algorithms were only applied on the training set to train a better model on the balanced dataset.

RETRACTED

To eliminate the influence of the dimension and order of magnitude and to ensure the reliability of the results, *Z* score standardization and mean standardization were performed on the training set to learn its parameters, and then the parameters were applied to the test set to normalize the data. The data were processed by principal component analysis or Pearson's correlation coefficient. The principal component analysis deleted the closely related and repetitive variables and established as few new variables as possible so that the new variables were irrelevant. Pearson's correlation coefficient was used to evaluate the linear correlation of the data. If the PCC value of both features was greater than 0.99, one was removed. After this process, the dimension of the feature space was reduced, and each feature was independent of the others.

The recursive feature elimination method or the Kruskal-Wallis test was used to select the features. Recursive feature elimination was used to filter out the best features through repeated construction of the model, and this process was repeated until all features were involved. The Kruskal-Wallis test was used to determine the relationship between the features and labels. The features were sorted according to the corresponding value, and the first 20 features were selected based on the validation performance.

### 2.5. Model Building and Model Validation

All models (including the *T*1 model, *T*2 model, and *T*1 + *T*2 model) were constructed by a multivariate logistic regression algorithm, and we used 5-fold cross-validation to obtain a stable and reliable model. The multivariate logistic regression model was a linear classifier that combined all of the features, and this model described the role of the various factors compared with the reference classification. Finally, a receiver operating characteristic (ROC) curve was drawn, and the area under the curve (AUC) and accuracy (ACC) were calculated for quantitative analysis.

We calculated the radiomics feature score by multivariate logistic regression analysis. The age and gender of the patients were considered potential predictors and were combined with the radiomic features to construct a nomogram for predicting postoperative recurrence and pseudoprogression of gliomas. As a visual tool, this nomogram provides clinicians with a quantitative tool to distinguish postoperative recurrence and pseudoprogression of gliomas, and this nomogram can help to guide clinical decision-making. In addition, a calibration curve was constructed, and the Hosmer-Lemeshow test was used to evaluate the nomogram of the training group and the testing group. To reflect the obvious incremental utility of the radiomic features, the clinical effectiveness was evaluated using the *T*1 model, *T*2 model, and *T*1 + *T*2 model to construct a decision curve analysis.

RETRACTED

### 2.6. Statistical Analysis

FAE software (https://github.com/salan668/FAE) was used for feature extraction, feature selection, and model construction. The data processing and statistical analysis were performed using SPSS software, version 26.0, and R software (http://www.R-project.org). All statistical tests were two sided, and the difference was considered statistically significant if *P* < 0.05.

## 3. Results

A total of 1316 features were extracted from the T1WI-CE and T2-FLAIR images in each patient, including 108 first-order intensity features, 14 shape features, 144 gray-level cooccurrence matrix (GLCM), 96 gray-level run length matrix (GLRLM), 96 gray-level size zone matrix (GLSZM), 30 neighborhood gray-tone difference matrix (NGTDM), 84 gray-level dependence matrix (GLDM), and 744 wavelet features. There were 2632 radiomic features in each patient. The process and results of feature selection and model construction are shown in Figure 6. The positive and negative samples in the dataset were balanced by the SMOTE algorithm, the *Z* score was standardized, the feature matrix was preprocessed by principal component analysis, and the features were selected using the recursive feature elimination method. Finally, 9 features were selected, and each PCA feature of the 118 patients is shown in Table 1. The *T*1 model was established by a multiple logistic regression algorithm. The AUC, ACC, sensitivity, and specificity of the training group were 0.815, 80.72%, 84.91%, and 73.33%, respectively. The AUC, ACC, sensitivity, and specificity of the test group were 0.804, 80.00%, 77.27%, and 84.62%, respectively. The ROC curve of the *T*1 model is presented in Figure 7. The SMOTE algorithm was used to balance the positive and negative samples in the dataset, the mean was standardized, Pearson's correlation coefficient was preprocessed to the feature matrix, and the Kruskal-Wallis test was used to select the features. Finally, 9 features were selected, and the *T*2 model was established by the multiple logistic regression algorithm. The AUC, ACC, sensitivity, and specificity of the training group were 0.754, 72.29%, 64.15%, and 86.67%, respectively. The AUC, ACC, sensitivity, and specificity of the test group were 0.734, 77.14%, 86.36%, and 61.54%, respectively. The ROC curve of the *T*2 model is presented in Figure 8. The 18 feature subsets of the *T*1 and *T*2 models were screened out, and the upsampling algorithm, mean standardization, and Pearson's correlation coefficient were used to preprocess the data. Then, the recursive feature elimination method was used to select the features, and the multiple logistic regression algorithm was used to establish the *T*1 + *T*2 model. The *T*1 + *T*2 model was composed of 12 features. The AUC, ACC, sensitivity, and specificity of the training group were 0.831, 77.11%, 75.47%, and 80.00%, respectively. The AUC, ACC, sensitivity, and specificity of the test group were 0.829, 88.57%, 95.45%, and 76.92%, respectively. The ROC curve of the *T*1 + *T*2 model is presented in Figure 9. The feature weight ranking diagrams of the *T*1 model, *T*2 model, and *T*1 + *T*2 model are shown in Figure 10. The features of the *T*1 model, *T*2 model, and *T*1 + *T*2 model, as well as the feature coefficients, are presented in Table 2. The PCA features constituting the *T*1 model are presented in Figure 11. The AUC, sensitivity, specificity, accuracy, positive predictive value, and negative predictive value of the *T*1 model, *T*2 model, and *T*1 + *T*2 model are presented in Table 3.

RETRACTED

The final results showed that the AUC values of the *T*1 + *T*2 model, *T*1 model, and *T*2 model in the training group were 0.831, 0.815, and 0.754, respectively, while those of the test group were 0.829, 0.804, and 0.734, respectively, indicating that the *T*1 model and *T*1 + *T*2 model showed good performance in the training group and test group. The prediction performance of the *T*1 + *T*2 model was better than that of the *T*1 or T2 model in both the training group and the test group. In addition, the sensitivity of the *T*1 + *T*2 model in the test group was better than that of the *T*1 or *T*2 model (95.45%, 77.27%, and 86.36%, respectively).

The radiomic nomograms in the training group and the test group are presented in Figures 12(a) and 12(b). The calibration curve of the nomogram shows that the discrimination probability was consistent with the actual occurrence in the training group. In the test group, the discrimination probability was roughly the same as the actual occurrence. The Hosmer-Lemeshow test showed that there was no significant difference (training group = 0.434, test group = 0.173), as shown in Figures 13(a) and 13(b).

With regard to decision curve analysis (DCA), the *T*1 + *T*2 model showed the highest overall net efficiency among the three models. When the threshold probability was between 0.15 and 0.30 and between 0.75 and 0.85, only the *T*1 model could achieve a higher net efficiency, as shown in Figure 14.

## 4. Discussion

An early diagnosis of recurrence and pseudoprogression of gliomas is challenging, and it is also difficult to individualize the comprehensive treatment to achieve the maximum therapeutic effect, to prolong the survival time and to improve the quality of life of patients. Currently, the common methods to diagnose recurrence and pseudoprogression of gliomas include conventional MR imaging, advanced MR imaging, and radiomics [15, 16]. Conventional MR imaging can only identify recurrence and pseudoprogression by imaging and clinical follow-up, delaying the timely adjustment of the treatment plan to a certain extent [17]. Compared with conventional MR imaging, advanced MR imaging has a certain value in distinguishing between recurrence and progression, but relying only on the parameter values of the local region of interest of the tumor is subjective. The image information mining is insufficient, and a single sequence cannot reflect the postoperative heterogeneity of the tumor tissue and the comprehensive information about the structural and functional changes [18]. In addition, partial advanced MR imaging (such as MRS and PWI) hinders the wide application of advanced MR imaging due to its relatively complex image acquisition and tedious postprocessing processes [19, 20]. For example, the results of MRS can be misleading because the spectra on the 3.0-T MRI scanner largely overlap with the rich brain metabolites, the spectral baseline is easily affected by substances such as blood, and these misleading results are very common in the postoperative treatment of gliomas [21]. However, some advanced MR imaging methods (such as ASL, DTI, and IVIM) are also hindered in their extensive clinical application because of their low spatial resolution and long scanning time [22–24]. Radiomics adopts computer image processing and big data mining methods, which can comprehensively evaluate the tumor characteristics, and it is helpful in devising a correct and detailed treatment plan and accurately evaluating the treatment effect. Therefore, the use of radiomics has important application value.

RETRACTED

This study was based on T2WI-FLAIR and T1WI-CE images to extract the imaging features. These sequences are relatively easy to obtain, are stable, and have been widely used in clinical practice. All levels and types of hospitals can achieve radiomics based on MRI, and the results are generally less affected by the differences in different types of MRI scanners. The results showed that, although pseudoprogression and recurrence have similar imaging findings, the different imaging features hidden in the images can be extracted and used to establish a correlation prediction model to distinguish between the two with relatively high reliability. Kim et al. [25] reported that T1WI-CE, T2WI-FLAIR, ADC, and CBV images of 61 patients with glioblastomas (35 cases of recurrence and 26 cases of pseudoprogression) in the early stage of radiotherapy and chemotherapy could be analyzed by radiomics. A total of 6472 radiomic features were extracted in that study. It found that a radiomics analysis of conventional MRI imaging combined with diffusion and perfusion imaging could better predict early recurrence and pseudoprogression, and the predictive efficiency was better than that of a single MRI sequence model (AUC = 0.90/0.85). Our study showed that, for the *T*1 + *T*2 model (that is, the multiple logistic regression model based on the T1WI-CE and T2WI-FLAIR sequences), the AUC of the training group was 0.831, and the AUC of the test group was 0.829, which was better than that of the single sequence model (*T*1 model and *T*2 model). The results are consistent with the above reports, and these results provide strong support for the use of these models for an accurate and timely diagnosis, improving the treatment of postoperative gliomas. In addition, Elshafeey et al. [26] analyzed the DSC-MRI and DCE-MRI images of 98 patients with glioblastomas in a three-center study (22 cases of pseudoprogression and 76 cases of recurrence). The radiomic features of rCBV and K^trans^ parameter images were extracted, and the classification model was constructed by SVM. It was found that the radiomics label of perfusion imaging can accurately predict the pseudoprogression and recurrence of glioma (ACC = 90.82%, AUC = 89.1%, sensitivity = 91.36%, and specificity = 88.24%). Compared with the results of our study, the diagnostic efficiency reported in the above literature was relatively higher, which could be because perfusion imaging can more accurately reflect the postoperative changes in gliomas. This modality provides a reliable alternative for the noninvasive identification of either pseudoprogression or recurrence. Sun et al. [27] retrospectively analyzed 77 patients with glioblastomas confirmed by surgical pathology. Based on the T1WI-CE sequence, the enhanced part was delimited as the region of interest, 9675 features were extracted, and a random forest (RF) classifier was used to establish a model to distinguish recurrence from pseudoprogression. Studies have shown that the performance of the T1WI-CE imaging model in the diagnosis of either recurrence or pseudoprogression of glioblastoma is relatively high. This study showed that the *T*1 model, that is, the multiple logistic regression model based on the T1WI-CE sequence, had an AUC of 0.815, sensitivity of 84.91%, specificity of 73.33%, and accuracy of 80.72%. In the test group, the AUC was 0.804, the sensitivity was 77.27%, the specificity was 84.62%, and the accuracy was 80.0%. The diagnostic efficiency of our study was higher than that of the above literature. The reason might be that the sample size of this study was relatively large, and different classifiers were used to establish the model. Therefore, this model could help clinicians to formulate an appropriate treatment plan as soon as possible.

RETRACTED

The above studies showed that the combined model (*T*1 + *T*2 model) is the most effective in predicting recurrence and pseudoprogression of gliomas, followed by the T1WI-CE model (*T*1 model). The conclusions of the study are basically consistent with the report of Gao et al. [28], so this study has important clinical application value. Moreover, this study performed decision curve analysis. Among the three models, the *T*1 + *T*2 model had higher overall net efficiency, but when the threshold probability was between 0.15 and 0.30 and between 0.75 and 0.85, only the *T*1 model obtained higher net efficiency, which has rarely been reported in previous studies [29], providing a new idea and method for the postoperative clinical diagnosis and treatment of gliomas in the future.

Previous studies have extracted features from MRI sequences and PET images and have established classifier models to predict recurrence and pseudoprogression in gliomas. Although these studies have achieved good results, they have also had some shortcomings. First, the number of samples in these studies was relatively small, and the proportion of patients with recurrence and pseudoprogression in these studies was unbalanced, affecting the accuracy of the results [30]. Second, the imaging techniques, particularly the techniques that use some advanced MR imaging, have higher equipment requirements, have more complex image acquisition, and require the use of tedious postprocessing software, so it is difficult to achieve in some grassroots hospitals [31]. Of course, this study also has some limitations. (1) It was a retrospective analysis, and the sample size was also relatively small. (2) A pathological examination is an invasive examination, and only a small number of confirmed cases were included in this study. Therefore, in this study, most patients were diagnosed based on a long-term follow-up longer than 6 months, and some patients were lost to follow-up. (3) There was no exact standard for tumor ROI segmentation, and the tumor edge could become blurred due to the local volume effect. Therefore, the tumor edge sometimes could not be determined accurately on the medical images. Moreover, this process is time consuming, and a more in-depth assessment of the variability and stability of the extracted imaging features between the patients is needed. In addition, as a retrospective study, the roles of molecular and genetic features, such as MGMT methylation and IDH1/2 mutation, were not evaluated in this study. It was reported that these molecular markers play an important role in the treatment of gliomas [32–34]. As a retrospective study, the role of clinical features, such as WHO grade, treatment after surgery, and perifocal edema, was not involved in this study. It was reported that these features play an important role in the postoperative evaluation of glioma [35–37]. (4) Due to the heterogeneity of gliomas after treatment, the results of pathology from a biopsy could have led to false negative results. No rigorous point-to-point pathological validation studies were performed in this study. Therefore, as a next step, it is necessary to increase the sample size and conduct further research on related molecular markers to render the results more reliable and to increase the diagnostic efficiency. (5) The radiomics model will be tested using other machine learning algorithms in our future study, for example, the enhanced *k*-NN algorithm [38], SVM [39], or tree-based classifier [40].

RETRACTED

## 5. Conclusion

In conclusion, multimodal MRI radiomic models based on T2WI-FLAIR and T1WI-CE images could predict postoperative recurrence and pseudoprogression of gliomas early, and this model could help clinicians to devise correct treatment plans so that patients can receive timely and accurate treatment, with important clinical value.

## Figures and Tables

**Figure 1:** A flowchart of the radiomics process for the prediction of recurrence and pseudoprogression of glioma.

**Figure 2:** Patient, male, 50 years old, left parietal lobe glioblastoma. (a) shows the T2WI-FLAIR scanning image before the operation; (b) shows the T1W1-CE scanning image before the operation; (c) shows the T2W1-FLAIR scanning image 1 day after the operation; (d) shows the T1W1-CE scanning image 1 day after the operation; (e) shows the T2WI-FLAIR scanning image 2 months after synchronous radiotherapy and chemotherapy; (f) shows the T1WI-CE scanning image 2 months after synchronous radiotherapy and chemotherapy; (g) shows the histopathological results (HE ×40) of the lesion removed during the second operation, which confirmed the recurrence of glioblastoma; (h) shows the T2WI-FLAIR ROI segmentation image 2 months after synchronous radiotherapy and chemotherapy; (i) shows the T1WI-CE ROI segmentation image 2 months after synchronous radiotherapy and chemotherapy.

**Figure 3:** Patient, male, 70 years old, left frontal lobe glioblastoma. (a) shows the preoperative T2WI-FLAIR scanning image; (b) shows the preoperative T1WI-CE scanning image; (c) shows the T2W1-FLAIR scanning image 1 day after the operation; (d) shows the T1W1-CE scanning image 1 day after the operation; (e) shows the T2WI-FLAIR scanning image 3 months after synchronous radiotherapy and chemotherapy; (f) shows the T1WI-CE scanning image 3 months after synchronous radiotherapy and chemotherapy; (g) shows the T2WI-FLAIR scanning image 11 months after synchronous radiotherapy and chemotherapy; (h) shows the T1WI-CE scanning image 11 months after synchronous radiotherapy and chemotherapy. The enhancement range of the lesion was reduced, confirming pseudoprogression. (i) shows the T2WI-FLAIR ROI image after 3 months of synchronous radiotherapy and chemotherapy; (j) shows the T1WI-CE ROI image after 3 months of synchronous radiotherapy and chemotherapy.

RETRACTED

**Figure 4:** Patient, male, 65 years old, left parietal lobe astrocytoma (WHO III). (a) shows the T2WI-FLAIR scanning image before the operation; (b) shows the T1W1-CE scanning image before the operation; (c) shows the T2W1-FLAIR scanning image 1 day after the operation; (d) shows the T1W1-CE scanning image 1 day after the operation; (e) shows the T2WI-FLAIR scanning image after 1 month of synchronous radiotherapy and chemotherapy; (f) shows the T1WI-CE scanning image after 1 month of synchronous radiotherapy and chemotherapy; (g) shows the histopathological results (HE ×100) of the second operation, confirming pseudoprogression; (h) shows the T2WI-FLAIR ROI image after 1 month of synchronous radiotherapy and chemotherapy; (i) shows the T1WI-CE ROI image after 1 month of synchronous radiotherapy and chemotherapy.

**Figure 5:** Patient, female, 47 years old, left frontal lobe glioblastoma. (a) shows the preoperative T2WI-FLAIR scanning image; (b) shows the preoperative T1WI-CE scanning image; (c) shows the T2W1-FLAIR scanning image 1 day after the operation; (d) shows the T1W1-CE scanning image 1 day after the operation; (e) shows the follow-up T2WI-FLAIR scanning image 2 months after the synchronous radiotherapy and chemotherapy; (f) shows the follow-up T1WI-CE scanning image 2 months after the synchronous radiotherapy and chemotherapy; (g) shows the follow-up T2WI-FLAIR scanning image 9 months after the synchronous radiotherapy and chemotherapy; (h) shows the follow-up T1WI-CE scanning image 9 months after the synchronous radiotherapy and chemotherapy, confirming recurrence. (i) shows the T2WI-FLAIR ROI image after 2 months of synchronous radiotherapy and chemotherapy; (j) shows the T1WI-CE ROI image after 2 months of synchronous radiotherapy and chemotherapy.

**Figure 6:** Process of feature selection and model construction.

RETRACTED

**Figure 7:** The ROC curve of the *T*1 model.

**Figure 8:** The ROC curve of the *T*2 model.

**Figure 9:** The ROC curve of the *T*1 + *T*2 model.

**Figure 10:** Feature weight ranking diagram of the *T*1 model, *T*2 model, and *T*1 + *T*2 model.

**Figure 11:** The PCA features constituting the *T*1 model.

**Figure 12:** (a, b) show the nomogram of the *T*1 + *T*2 model in the training group and test group, and the model included sex, age, and radiomics features. The “risk” represents the risk of tumor recurrence.

**Figure 13:** (a, b) are the calibration curves of nomogram of the training group and the test group, respectively. (a) is the calibration curve of nomogram of the training group, and the result was insignificant based on the Hosmer-Lemeshow test (*P* = 0.434). (b) is the calibration curve of nomogram of the test group, Hosmer-Lemeshow test (*P* = 0.173). “Ideal” is the standard curve, “apparent” is the prediction curve, and “bias-corrected” is the prediction curve of validation, showing the actual performance of the nomogram.

**Figure 14:** Represents decision curve analysis (DCA). The net benefit is plotted on the *y*-axis, and the high-risk threshold is plotted on the *x*-axis. The solid black line assumes that not all patients with gliomas experience recurrence and do not receive treatment. The solid gray line assumes that all patients with gliomas have recurrence and receive treatment. The red line represents the *T*1 model, the blue line represents the *T*2 model, and the yellow line represents the *T*1 + *T*2 model.

**Table 1:** Each PCA feature of the 118 patients constituting the *T*1 model.

PCA_feature_4	PCA_feature_5	PCA_feature_16	PCA_feature_21	PCA_feature_29	PCA_feature_46	PCA_feature_70	PCA_feature_75	PCA_feature_84
5.292285	-0.31922	-4.00436	-1.98362	0.533162	-2.27227	1.130868	0.420055	4.66E-15
47.39251	3.492607	-0.23689	1.808537	-0.36735	-0.44124	-0.02491	-0.05254	1.91E-14
14.02842	29.67719	9.214032	-4.79484	0.075233	-0.23415	-0.02585	0.122281	-6.72E-15
9.34525	-9.15225	-1.21241	4.839331	-0.57513	0.299695	-0.89978	0.740213	9.06E-15
-6.52724	-2.08316	2.517063	-0.33012	1.305346	-0.46286	0.182298	0.145839	3.00E-15
78.68403	106.741	48.92409	-39.1934	78.42099	-30.303	-45.5879	42.08611	-7.974691577
2.616511	-2.10086	-1.17164	-0.36293	0.322589	2.183477	0.822964	0.170237	-9.89E-15
0.4149	15.44613	-4.93932	2.242049	-0.65424	0.095358	-0.07338	5.264379	-0.439794471
14.07457	0.470138	-17.9888	6.244064	6.404484	-3.82665	-0.48285	-1.64905	0.664957879
-2.32219	3.0981	-2.43291	-1.45249	0.678227	-0.00956	-1.09041	-0.01811	4.15E-15
3.217888	5.469739	-2.18855	-4.3385	0.679512	1.797729	0.030073	0.313115	1.94E-16
-0.65419	2.731624	-0.9656	1.97338	-1.78015	0.853095	0.084391	-0.0887	-2.11E-15
-6.80974	-0.24792	-6.85001	2.125862	2.759247	-1.488	-0.24255	0.15168	-1.66E-15
5.948918	-0.51271	-5.42461	2.62764	-2.35276	1.426647	-0.30227	-0.56675	0.065632207
-0.93126	-3.31027	0.524146	-0.70658	3.144197	1.40874	-0.25546	1.114749	0.119017488
-4.25023	-7.30925	1.059886	-4.34909	2.98548	2.959464	-0.3118	-0.10746	-2.28E-15
18.65532	-6.25942	4.936938	-4.57648	-3.71226	0.02198	-0.21541	0.042243	1.66E-14
-10.0307	37.23263	-12.4094	8.17473	-2.7618	-11.9517	-9.15899	1.715302	-1.394932254
-6.81928	24.40381	-7.72651	3.244765	-3.19724	-0.39126	-0.19786	0.057621	-6.16E-15
1.01572	-1.81784	-2.92512	-2.18604	-0.04629	0.697968	-1.07247	-0.69389	-1.41E-14
-13.5146	0.184732	-0.77833	-0.90736	1.462477	0.005882	-0.07868	1.653141	0.039443876
-0.022	-6.93584	1.53938	1.994829	4.44277	-1.10635	0.63898	-0.41743	9.54E-15
7.71877	-2.19661	0.596954	0.722368	-2.10545	-0.06838	-0.49699	-0.2902	3.23E-15
-0.2804	-6.65688	-0.59073	-1.53381	-0.50513	0.916167	0.450793	-0.16584	1.26E-15
-3.24134	0.01103	0.217441	1.683541	-1.71613	-0.25424	-0.33535	0.209327	-0.280006287
-4.74777	-6.59527	4.367952	-1.85506	1.263532	-1.33841	-0.29556	0.865688	-3.26E-15
-15.1729	-1.63566	-3.20933	-4.31179	3.885077	1.422653	0.277829	-0.02723	1.28E-15
6.07457	11.39398	-5.63322	-6.7955	1.532886	-0.56114	0.283856	0.026022	1.04E-14
-5.21004	-3.17045	-0.99247	-0.64768	0.57616	-0.8578	-0.3636	-0.59327	-2.71E-16
0.636277	-4.44734	-0.61923	2.55714	2.683026	-0.50991	-0.97375	-0.4067	-3.41E-15
1.811859	9.254191	0.141253	4.858761	-2.01516	-0.10016	2.29529	-0.03757	2.03E-15
-2.79984	2.170599	0.145647	1.711067	-0.93871	-0.149	1.355029	0.616871	0.238106924
-10.3766	-2.58322	-3.35344	-1.46963	-4.46713	-0.8258	-0.15446	-0.03716	6.72E-15
0.521226	0.893289	-7.2868	5.764718	1.606701	-1.82732	-0.18693	-0.17211	3.07E-15
-3.30438	-4.11744	-0.49157	-0.87634	-0.04762	0.029446	-0.7039	0.152189	-0.086473796
9.037669	-6.11028	-2.67521	-1.0285	-1.35297	-0.11059	0.831632	0.143292	4.82E-15
7.413207	12.54606	-1.82201	-3.80765	1.301612	1.021206	-1.13343	-0.34302	-2.94E-15
-2.14979	2.400672	-2.94575	-0.28709	1.340684	-2.00597	1.387555	-0.46184	2.91E-15
-4.74829	14.68956	-6.38626	-4.55795	7.202112	0.835627	-0.12122	1.316051	-1.040748763
8.63982	-1.03431	-5.57777	-3.31887	-2.12002	0.774806	0.051979	-0.04307	-3.96E-16
-3.79514	0.881233	-0.94252	2.247918	1.840978	0.108199	-0.63709	-0.71274	0.232555979
2.399948	9.46091	-5.58438	-1.44095	-1.72839	0.286107	0.016429	0.029347	-1.27E-14
-1.5997	1.624524	0.119268	0.399976	1.050154	-1.03302	-2.23905	1.705516	6.11E-16
3.829345	-2.56345	1.340711	1.067721	1.394663	0.844944	-0.84952	-0.20728	-8.30E-15
-3.39658	2.919978	-2.40053	-0.95138	-2.27651	-2.54432	-0.2426	0.221639	1.24E-15
9.069545	-0.8728	-3.30846	-0.81162	0.671909	0.166787	-0.6071	1.059451	-0.353128638
5.926697	-4.44445	-0.52153	1.970514	-1.75058	-1.50587	0.164515	-0.66155	-0.028937381
-8.81656	-4.51862	3.884953	-1.85198	-3.43412	-1.20734	-0.26332	0.047992	2.98E-16
3.403512	8.876643	-3.32883	6.130056	-3.3399	0.951617	-1.18803	-0.84505	-7.36E-15
1.02342	-3.263	-0.06198	-1.33908	0.656886	1.025216	-1.13782	-1.25926	-5.90E-16
0.991009	3.089894	-3.12464	-1.12885	2.207428	0.585581	0.911663	0.104456	-5.25E-15
-1.5018	4.460188	-3.16622	1.711252	-0.44877	-0.31562	0.676643	-0.2555	-3.26E-15
21.49179	22.71561	-0.98575	-6.7607	10.88672	-5.73668	-2.65564	6.287265	-0.160435432
8.146266	-10.3074	-0.0662	-1.22035	1.09751	0.634754	-0.13256	0.867994	-1.31E-14
-4.44646	-3.29724	-1.2867	1.531712	2.24025	2.535474	0.01643	0.582372	-4.77E-15
8.897867	15.01368	-0.10585	-4.03512	3.660932	1.495116	-0.21596	1.484205	-0.19507939
1.724314	-4.96044	0.372722	1.405166	-1.08415	-0.00081	1.740313	0.648018	5.11E-15
-3.34509	-2.71972	-1.27086	0.631356	2.143476	0.641056	-1.08643	-0.74238	0.369842752
0.004694	-1.79716	1.693811	10.93441	2.130789	-0.13781	-0.11229	-0.0259	1.13E-14
-0.93755	8.695374	3.832587	1.428436	0.482639	-0.46109	0.162263	-0.17125	-7.49E-16
3.799824	-0.24524	2.026396	0.880298	1.668643	-1.33702	-0.26365	0.623905	0.300475474
-1.02919	0.469794	-3.4455	1.109414	-0.4014	0.262985	0.429931	1.204178	-1.36E-15
0.537844	-1.84696	-1.14815	2.444493	0.83327	0.515927	-0.45877	-0.18453	-7.09E-15
-6.02878	6.081398	0.432533	0.157935	-0.42553	-0.36609	0.053607	0.045802	-2.74E-15
43.92076	-1.07085	6.317528	-8.70503	12.65221	1.622631	10.0393	-3.24109	-4.218612815
0.07159	-3.04047	3.770569	0.762228	-0.47138	1.501355	-0.10714	1.499657	-5.55E-17
15.43612	18.24185	9.928053	7.710709	-4.53731	0.505533	-2.87046	-2.69788	-0.628829234
0.421393	0.039008	1.563885	0.323148	1.381905	0.95794	0.161991	-0.1396	-8.62E-15
-5.20541	-3.51989	3.498475	0.076886	2.276971	-0.66577	0.250564	-0.32387	2.60E-15
-4.0874	13.87052	-9.60037	-1.03243	-0.14495	0.318006	-1.43098	1.960888	-0.698018074
-5.24155	-5.08264	-0.6336	-2.23368	-1.28038	-0.55043	0.288405	-0.54143	1.17E-15
-2.64837	13.33802	1.000848	5.880341	1.079573	1.983298	-0.34444	0.188482	-7.91E-16
-2.37035	6.564671	2.046507	0.381795	-2.04302	-1.27837	-0.44826	-0.74171	-1.19E-15
-0.85353	-5.24516	2.462755	-2.84822	-1.45034	-1.46855	-0.08318	-0.04062	7.22E-16
-1.06877	-2.60263	-0.27898	-1.32775	0.41865	-0.06679	-0.44401	1.457391	-4.84E-15
-1.83821	4.44197	-0.68852	-3.49756	0.778103	0.982541	1.502637	0.281243	-0.167778149
6.960689	8.371046	4.511933	4.073733	-0.32784	1.050152	0.061903	-0.02172	-2.14E-15
109.7929	92.97725	5.275556	-59.681	65.70477	-65.3376	-28.7198	52.72077	-2.353897398
-4.69332	26.10232	-7.25716	-3.98726	5.232468	5.286849	3.377791	0.465964	-0.301807389
32.21627	-23.9823	-0.37751	-0.16022	1.411639	0.151863	0.112674	-0.23666	1.41E-14
-10.966	3.04883	-0.59678	0.895091	-0.61039	1.702601	0.055435	0.333552	0.158601857
-20.8874	12.49018	-5.3943	-2.15856	4.927952	-0.89899	-0.33394	-0.05387	-1.90E-14
-11.1189	23.44627	6.519808	-1.69246	1.088536	0.985096	0.215908	0.044966	-5.55E-16
12.72998	-8.36748	-7.73686	4.6243	4.253367	-1.97772	0.339672	0.154623	7.36E-15
-13.3721	-5.20197	4.701933	-0.5775	0.412411	0.3186	-0.20103	0.225601	-2.14E-15
12.56204	16.08144	-3.63944	-5.01474	2.467282	-2.46295	0.216706	0.175155	1.18E-14
2.699453	0.072194	7.416495	2.396091	-3.55825	-2.23968	0.235043	0.012939	-7.77E-15
-0.3861	-4.76557	2.105854	-0.92855	3.240122	-0.22599	-0.74138	-0.7086	0.19120143
-11.8926	-3.12207	-3.1087	0.236522	-3.06119	3.745754	0.772919	-0.61883	3.57E-15
22.41741	14.69678	0.138025	2.495278	1.990452	-4.6134	-6.83481	-1.71435	-0.911812617
-3.18317	1.39274	-1.17846	0.756758	-2.11342	-0.19189	0.389699	2.266525	1.14E-15
33.62059	-5.18131	14.83547	-7.23177	-2.61357	7.698903	2.862415	-1.1364	0.211704815
1.870208	-4.31568	-0.23749	0.721528	1.012697	1.038231	0.353299	-0.09122	1.71E-15
-13.1781	-9.73399	-1.30941	-0.26797	-3.73141	-3.24848	-1.25447	0.400919	-1.25E-14
1.576719	-3.60685	-2.11557	-1.33998	-0.57935	-2.33651	-0.01277	-1.4884	-0.210243395
1.493117	-6.27215	0.962873	-0.39145	0.336636	0.055183	0.083143	-1.17633	-3.29E-15
-4.47393	-9.35485	-0.88192	-1.01499	-3.30139	3.153677	0.060731	0.689323	3.79E-15
1.477406	-7.54656	-1.97466	-0.98841	-0.18062	2.412202	-1.09157	0.720796	-8.26E-16
2.494601	-3.77051	1.102043	0.071758	0.943959	-0.96403	-0.79065	0.768234	2.64E-16
2.392249	-7.33487	9.024553	1.589005	2.740353	-1.17782	0.201953	0.032109	8.77E-15
-9.98714	-7.77169	3.302531	0.659957	0.396025	-0.06744	1.273564	0.094813	-5.00E-15
-2.20105	10.06914	1.850717	4.478965	-1.47993	-0.98854	0.252559	-0.17416	-2.57E-15
6.737719	9.565899	1.866756	3.552694	3.806825	-0.11602	-0.15844	0.054108	4.87E-15
-0.96119	-8.57707	1.537709	-0.71854	0.401047	0.991741	0.720644	-0.35734	0.578490314
-1.83948	-1.86587	-0.12682	-2.63646	0.696986	0.693659	0.790789	-0.17537	-1.71E-15
1.72582	-6.47299	-2.48477	-0.42839	-0.91825	-0.74634	-1.33064	-0.46122	-3.29E-15
-6.92553	9.055262	1.850103	3.102281	-2.03538	1.510992	-0.52105	-0.11016	1.73E-15
-3.81024	1.986353	4.2684	3.151188	0.371766	0.475246	-0.42689	-0.05438	-1.70E-15
17.36278	20.23298	3.612801	-2.772	-0.79898	0.230551	-0.07971	0.069878	-1.80E-14
1.815338	-0.44389	-1.67253	0.663319	-3.16097	0.566102	1.058888	-0.30745	5.01E-15
-9.07824	9.699117	-6.285	-6.37076	8.140719	5.631762	1.387593	-1.4395	0.187102481
0.511153	-7.02786	-0.78138	1.23305	-2.53651	0.900582	1.339958	1.497985	0.740895249
-2.05504	-2.71125	-1.54173	-0.61195	3.702956	0.21079	-1.20309	1.09066	0.026452611
-3.36717	0.612464	0.416177	3.081299	1.231177	2.327259	-0.16466	0.030477	-6.86E-15
-9.13871	-8.35627	-1.96923	1.444825	-0.90834	2.632397	-0.67799	0.194453	-0.113946114
3.420181	5.388643	1.914437	-3.06878	2.955113	1.764999	0.047246	-0.08285	-1.54E-14
138.7889	-23.2254	45.52179	-38.3533	-34.3425	39.0107	-9.84405	-5.43453	-5.167926593
1.386581	-5.47372	2.112693	0.900384	-1.16614	0.346788	-0.63855	-1.42455	1.45E-15

RETRACTED

**Table 2:** Features and feature coefficients of the *T*1 model, *T*2 model, and *T*1 + *T*2 model.

	Features	Coeff. in model
*T*1 model	PCA_feature_4	0.071414853
	PCA_feature_5	0.085357498
	PCA_feature_16	-0.126573226
	PCA_feature_21	0.209233438
	PCA_feature_29	0.343369903
	PCA_feature_46	0.416733598
	PCA_feature_70	-0.274741275
	PCA_feature_75	0.197216124
	PCA_feature_84	-2.94E-15
*T*2 model	T2FLAIR_wavelet-HHH_firstorder_Kurtosis	-0.718270276
	T2FLAIR_wavelet-HHL_firstorder_Kurtosis	-2.304664815
	T2FLAIR_wavelet-HHL_glszm_GrayLevelNonUniformityNormalized	-0.716046488
	T2FLAIR_wavelet-HHL_glszm_GrayLevelVariance	1.059426151
	T2FLAIR_wavelet-HLL_glszm_GrayLevelNonUniformityNormalized	-2.641634777
	T2FLAIR_wavelet-HLL_glszm_SmallAreaEmphasis	2.697093602
	T2FLAIR_wavelet-LHL_glcm_Id	0.442493485
	T2FLAIR_wavelet-LHL_glcm_Imc1	2.913271424
	T2FLAIR_wavelet-LHL_glcm_InverseVariance	-2.791086243
*T*1 + *T*2 model	PCA_feature_5	4.599393961
	PCA_feature_21	2.326570486
	PCA_feature_29	4.309198531
	PCA_feature_46	8.818934434
	PCA_feature_70	-9.605827649
	PCA_feature_75	8.114281221
	T2FLAIR_wavelet-HHH_firstorder_Kurtosis	-0.967832041
	T2FLAIR_wavelet-HLL_glszm_GrayLevelNonUniformityNormalized	-2.334267326
	T2FLAIR_wavelet-HLL_glszm_SmallAreaEmphasis	1.942247316
	T2FLAIR_wavelet-LHL_glcm_Id	-2.50250236
	T2FLAIR_wavelet-LHL_glcm_Imc1	0.393741775
	T2FLAIR_wavelet-LHL_glcm_InverseVariance	-2.552759027

**Table 3:** Diagnostic effectiveness of the *T*1 model, *T*2 model, and *T*1 + *T*2 model.

Model type	Training group						Test group					
	AUC	Accuracy	Sensitivity	Specificity	PPV	NPV	AUC	Accuracy	Sensitivity	Specificity	PPV	NPV
*T*1 model	0.815	80.72	84.91	73.33	84.91	73.33	0.804	80.00	77.27	84.62	89.47	68.75
*T*2 model	0.754	72.29	64.15	86.67	89.47	57.78	0.734	77.14	86.36	61.54	79.17	72.73
*T*1 + *T*2 model	0.831	77.11	75.47	80.00	86.96	64.86	0.829	88.57	95.45	76.92	87.57	90.91

## Data Availability

The datasets used and/or analyzed during the current study are available from the corresponding author on reasonable request.
